This article has been retracted.

# Sufentanil alleviates pre-eclampsia via silencing microRNA-24-3p to target 11β-Hydroxysteroid dehydrogenase type 2

**DOI:** 10.1080/21655979.2022.2066753

**Published:** 2022-05-04

**Authors:** Yang Yue, Fu Xu, JiaRong Zhang, Miao Zhao, FangFang Zhou

**Affiliations:** a Department of Obstetrics, Longhua District Maternity and Child Health Hospital, Shenzhen, Guangdong, China; b Department of Anesthesiology, Longhua District People’s Hospital, Shenzhen, Guangdong, China

**Keywords:** HTR8/SVneo cells, preeclampsia, trophoblast, Sufentanil, 11β-hydroxysteroid dehydrogenase type 2

## Abstract

Pre-eclampsia (PE) is a prevalent pregnancy disease characterized by insufficient trophoblast cell migration (HTR8/SVneo). Consequently, accelerating trophoblast cell proliferation might ameliorate PE. This study assessed the effects and molecular mechanisms of Sufentanil (SUF) on HTR8/SVneo cells proliferation. HTR8/SVneo cells and PE clinical samples were used. Peripheral blood was collected from PE patients’ samples, and microRNA (miR)-24-3p and 11β-hydroxysteroid dehydrogenase type 2 (HSD11B2) was analyzed in the blood and cells. HTR8/SVneo cells were treated with varying SUF concentrations or transfected with miR-24-3p mimics/inhibitors, or HSD11B2 elevation vector. CCK-8, colony formation, transwell, and flow cytometry assays were then carried out. Association of miR-24 − 3p with HSD11B2 was investigated. PE animal model was constructed using Wistar rats to verify SUF’s role on PE *in vivo*. According to the results, SUF boosted HTR8/SVneo cell proliferation, and inhibited miR-24-3p to accelerate HSD11B2. MiR-24-3p was increased in PE, while HSD11B2 was inhibited, and miR-24-3p targeted HSD11B2. HSD11B2 reversed miR-24-3p’s repression on HTR/SVneo cell advancement. SUF restrained PE’s progression in *vivo* and in *vitro* via mediating the miR-24-3p/HSD11B2 axis. In conclusion, SUF enhances HSD11B2 via repressing miR-24-3p, thereby suppressing PE’s progression. The study provides an insight into the possibility of using SUF as a novel therapeutic target for PE, which acts via combining with miR-24-3p.

## Highlights

- SUF accelerated HTR8/SVneo cell proliferation.
- MiR-24-3p inhibited HTR8/SVneo cell progression.
- MiR-24-3p targeted HSD11B2 in PE.
- HSD11B2 reverses the miR-24-3p suppressor effect on HTR8/SVneo cell growth.
- SUF down-regulated PE progression in vivo via miR-24-3p/HSD11B2 axis.

## 1 Introduction

Pre-eclampsia (PE) is a hypertensive disorder complicating pregnancy, impacting 2% to 8% of pregnancies worldwide and leading to distinct maternal and perinatal morbidity and mortality [1]. Several studies have investigated the pathophysiological mechanisms of PE, but the precise pathogenesis of PE remains unclear [2]. Additionally, safe and imperative PE therapy and biomarkers for early diagnosis have not been developed [3]. Presently, reports have clarified that the incidence of PE is associated with trophoblast dysfunction [4]. Nevertheless, the regulatory mechanism of trophoblast invasiveness remains uncertain.

Sufentanil (SUF) is a widely adopted opioid, appropriate for moderate and severe acute pain from intravenous and intrathecal treatment due to the absence of active metabolites [5]. Anesthesia can not only restrain the stress response caused via surgery and pain but also directly or indirectly impact the cell function after surgery [6]. According to various studies, SUF has a protective role in different diseases via modulating microRNA (miRNA). For instance, SUF preconditioning inhibits ischemia-reperfusion injury-stimulated oxidative stress and autophagy of myocardial cells via modulating miR-125a/damage-regulated autophagy modulator 2 axis [7]. SUF reduces ropivacaine-stimulated apoptosis of umbilical cord mesenchymal stem cells via mediating miR-182-5p/BCL10/CYCS axis [8]. Emerging research has also reported that SUF cures PE in combination with other drugs like long-term epidural analgesia (LTEA), naloxone, and Clonidine [9]. Nevertheless, the action of SUF alone in PE and its latent mechanism remain unknown.

MiRNA, a class of short endogenous non-coding RNA, modulates genes via repression or mRNA degradation after transcription, and it is implicated in the modulation of diversified biological processes, including cell growth and differentiation [10]. MiRNA are detected through various methods including nanomaterial-based techniques, nucleic acid amplification, and RCA-based techniques [11]. MiRNA, as the crucial mediator in biological processes, mediates about 60% of genes in eukaryotes, whose disorders are the reasons for various illnesses and are considered latent biomarkers and therapeutic targets for various diseases [12]. For instance, the role of miRNA in the progression of various cancers has been widely reported [13]. On reproductive health, considerable evidence has elucidated that aberrant miRNA leads to pregnancy complications like PE [12]. Additionally, miRNA regulates various cellular processes that maintain a healthy pregnancy, such as acceleration of angiogenesis and trophoblast cell differentiation [14]. MiR-24-3p, a broadly explored miRNA, is critical in gene modulation. Recent research confirmed that miR-24-3p is elevated in peripheral blood of PE patients, confirming that miR-24-3p might have a role in PE’s occurrence and development [15]. Nevertheless, the biological function of miR-24-3p in PE has not been investigated.

The study hypothesized that Sufentanil down-regulates the progression of pre-eclampsia via silencing microRNA-24-3p to target 11β-Hydroxysteroid Dehydrogenase Type 2 (HSD11B2). The study aimed to determine the effects of SUF on HTR8/SVneo cell viability, understand the effects of SUF on miR-24-3p and HTR8/SVneo cell proliferation, investigate the impacts of miR-24-3p mimicking on HTR8/SVneo cell progression, investigate if miR-24-3p targets HSD11B2 in PE and to understand the effects of SUF on HSD11B2 and HTR8/SVneo cell proliferation. Finally, the role of SUF in PE progression in vivo was investigated.

## 2 Experimental methods

### 2.1 Ethics statement

This study was authorized by the Ethics Committee of Longhua District Maternity and Child Health Hospital (Ethical approval number: LH-2016A3186). Written informed consent was obtained from all the study participants. The approved procedures were used for the humane treatment of animals following the National Institutes of Health Laboratory Animal Care and Use Guidelines recommendations.

### 2.2 Clinical specimens

From December 2019 to December 2020, 35 clinical samples were collected from Pre-eclampsia (PE) patients and pregnant women with normal blood pressure in Longhua District Maternity and Child Health Hospital. The average age was (28.50 ± 3.93) years, and the average gestational age was (34.15 ± 3.12) weeks. PE patients with systolic blood pressure ≥ 140 mm Hg (1 mm Hg = 0.133 kPa) at the first pregnancy, diastolic blood pressure ≥ 90 mm Hg and urine protein ≥ 0.3 g/d or random urine protein (+) and above after 20 weeks of pregnancy were selected. Within 24 h after delivery, 3 mL of peripheral blood was collected from each patient during the fasting period. After collecting the upper serum, the samples were centrifuged and stored in a dry and sterile Eppendorf (EP) tube for subsequent experiments [1].

### 2.3 Cell culture and transfections

The HTR8/SVneo cells were purchased from the American Type Culture Collection (ATCC; Manassas, VA, USA). The cells were cultured in Roswell Park Memorial Institute (RPMI)-1640 medium (Thermo Fisher Scientific, Waltham, USA) supplemented with 10% fetal bovine serum (FBS) (Thermo Fisher Scientific), 100 U/mL penicillin, and 100 mg/mL streptomycin. The cells were grown to a confluence of 70% and passaged for storage and subsequent assays.

For the transfection assay, the miR-24-3p mimics and inhibitors, corresponding negative control (NC), and HSD11B2 elevation vector was purchased from Guangzhou RiboBio Co., Ltd., (Guangzhou, China). Transfection of HTR8/SVneo cells was done using Lipofectamine 2000 (Invitrogen, CA, USA) according to the manufacturer’s instructions. The HTR8/SVneo cells were pretreated with 5, 10, 20 μM SUF (Yichang Renfu Pharmaceutical Co., Ltd., Yichang, China) [2].

### 2.4 Cell Counting Kit-8 (CCK-8) assay

The HTR8/SVneo cells (1 × 10^4^cells/mL) were plated in a 96-well plate and cultured for 24 h. After treatment with various concentrations of SUF and further culture for 24 hr, cell viability was determined by addition of 10 ul CCK-8 solution (Beyotime Biotechnology, Shanghai, China), according to the manufacturer’s instruction. The absorbance was finally measured at 450 nm was in a microplate reader (DU650, Beckman Coulter, CA, USA) OD450).

### 2.5 Colony formation assay

The HTR-8/SVneo cells from all the groups were harvested at the logarithmic phase, trypsinized, diluted, and counted under the microscope. Approximately 200 cells/ well were seeded in a 6-well plate and grown for 9 days. The medium was removed, and cells were fixed using 4% paraformaldehyde. The fixative was then discarded, and cells were stained for 1 h at room temperature using crystal violet. The cells were later washed, colony formation was determined under a fluorescent microscope, and colony numbers counted. The percentage rate of colony formation was calculated as colony number per 2 × 10^2^ cells × 100, as described elsewhere [16]. The experiment was done in triplicates.

### 2.6 Transwell assay

Cell invasion and migration were determined through the Transwell experiment as previously reported [17]. For the migration assay, a chamber of 8 μm pores (6.5 mm) (Corning Costar Corp., USA) was used. Approximately 2 × 10^4^ stably transfected HTR8/SVneo cells were resuspended in 200 μl of serum-free RPMI media and plated in the upper chamber. Later, the RPMI 1640 media (500 μl) supplemented with 10% fetal bovine serum was introduced in the lower well chamber. Cells were then incubated under the chemotactic condition at 37°C for 24 h.

The cells were stained for 30 min using 1% crystal violet, and cells on the membrane’s upper surface were removed using cotton swabs. The cells on the bottom of the membrane were quantified and imaged microscopically (Olympus Corp. Tokyo, Japan) in four random fields. For the invasion experiment, Matrigel, 0.1 ml (50 μg/ml, BD Biosciences, USA) was added to the plate and incubated for 2 h. The remaining assay steps were similar to the migration assay described above. The experiments were done in triplicate.

### 2.7 Flow cytometry detection

The apoptosis rate of HTR8/SVneo cells was done using flow cytometry and annexin V-fluorescein isothiocyanate (FITC)/propidium iodide (PI) (BD Biosciences, CA, USA) according to the manufacturer’s guidelines. In summary, after collecting HTR8/SVneo cells, the cells were incubated with 500 μL loading buffer, 5 μL Annexin V-FITC, and 10 μL PI solution as directed in Annexin-V-FITC Cell Apoptosis Detection Kit (Biovision, K101). The apoptosis rate was determined in a flow cytometer (BD Biosciences, Franklin Lakes, NJ, USA). The experiment was repeated three times, and the data were averaged.

### 2.8 Reverse transcription-quantitative polymerase chain reaction (RT-qPCR) analysis

Separation of total RNA was done using the TRIzol kit (Invitrogen). RNA concentration and purity were determined using Nanodrop 2000 (Thermo-fisher scientific). The reverse RNA transcription into complementary DNA (cDNA) was done using Prime Script™ RT-PCR kit (Takara Biomedical Technology, Dalian, China) following the manufacturer’s instructions. The RT-qPCR reaction system was done using SYBR Premix Ex Taq™ II (Takara Biomedical Technology) and Bio-Rad CFX-96 (Bio-Rad Laboratories, CA, USA). The glyceraldehyde 3-phosphate dehydrogenase (GAPDH) was used as an internal control. The results’ analysis was done using the 2^−ΔΔCt^ method. The primers were designed by Shanghai Shenggong Biotechnology Co., Ltd., (Shanghai, China). The primers are presented in Table 1.

**Table 1.** Primer sequences

Genes	Primer sequences (5’ – 3’)
MiR-24-3p	F: 5′-CGTGGCTCAGTTCAGCAG-3′
	R: 5′-GTCGTATCCAGTGCAGGGTCCGAGGTATTCGCACTGGATACGAC CTGTTC-3′
U6	F: 5’-CTCGCTTCGGCAGCACA-3’
	R: 5’-AACGCTTCACGAATTTGCGT-3’
HSD11B2	F: 5’-TCTAGAGTTCACCAAGGCCCA-3’
	R: 5’-GCAAGTGCTCGATGTAGTCCT-3’
GAPDH	F: 5′-CGACCACTTTGTCAAGCTCA-3′
	R: 5′- GGTTGAGCACAGGGTACTTTATT-3′

F, forward; R, reverse.

### 2.9 Western blot

After extracting PE embryo tissue or cells’ total protein, protein concentration was determined using the bicinchoninic acid protein quantitative kit (ThermoFisher Scientific). Proteins were separated with 10% sodium lauryl sulfate-polyacrylamide gel electrophoresis, and electroblot was transferred onto a nitrocellulose membrane. The membrane was blocked using 5% skimmed milk and incubated using primary antibodies HSD11B2 (1: 1000, ab203132), GAPDH (1 µg/mL, ab8245), and Immunoglobulin G (IgG) antibodies (1: 2000, ab97051) (Abcam, MA, USA).

The membranes were then incubated with the corresponding horseradish-conjugated secondary antibodies at room temperature for 1 h. Enhanced chemiluminescence solution (ECL808-25, Biomiga) was finally added to the membrane for color development. After scanning with a photometer (GE, Pittsburgh, USA), the protein bands were analyzed with Image-Pro Plus 6.0 software (Media Cybernetics, Silver Spring, Maryland, USA).

### 2.10 The luciferase activity assay

Prediction of the latent binding of miR-24-3p with HSD11B2 was made using the starbase website (http://starbase.sysu.edu.cn). The 3’-untranslated region sequence of HSD11B2 covering miR-24-3p wild-type (WT) or mutant (MUT) binding site was integrated into the pmirGLO vector (Promega, WI, USA) to form WT-HSD11B2 or MUT-HSD11B2. The miR-24-3p or mimic NC was then transfected into 293 T cells with Lipofectamine 2000 (Invitrogen) following the manufacturer’s protocol. Additionally, luciferase activity was determined through Dual-Luciferase Reporter Assay using Luciferase Reporter Kit (Promega).

### 2.11 RNA binding protein immunoprecipitation (RIP) assay

The Magna RNA Binding Protein Immunoprecipitation Kit (Merck KGaA, Darmstadt, Germany) was specifically designed for RIP analysis. Before performing the RIP assay, cells were lysed with RIP lysis buffer (Beyotime). Then, the cell lysates were incubated with magnetic beads conjugated with Argonaute-2 or control IgG (Millipore, MA, USA). The cells complex was detached using proteinase K (Sigma-Aldrich), and the identification of RNA binding was done using RT-qPCR.

### 2.12 Animal experiments

Adult Wistar rats (200 ± 20 g) were purchased from Jinan Experimental Animal Center (Shandong, China). After acclimatizing, the experimental rats were sustained at a 12-h light cycle, with free provision of standard rodent food and water. Male and female rats were kept together to allow for natural pregnancy in female rats. The following day after mating, wet cotton swabs were gently inserted into the female rat’s vagina; vaginal secretions were taken and smeared on a glass slide and observed under an optical microscope.

The presence of sperms in the vaginal smear manifested on the first day of pregnancy. The female rats were randomly divided into two groups at 1 week of pregnancy using a random number table, covering the normal pregnancy (the control) and the PE model. Rats in the PE group were subcutaneously injected with L-NAME 50 mg/kg at multiple places on the seven^th^ day of pregnancy to stimulate PE [3]. The control animals were injected with 0.9% normal saline of a similar dose. The treatments were repeated until the 11^th^ day of pregnancy. After constructing the PE model, the animals were divided into two subgroups: The PE and the SUF. Animals in the SUF group were intraperitoneally injected with SUF (5 μg/mL, 0.1 mL) once a day for three days [4]. The rats were euthanized after the 21^st^ day of pregnancy, and the placental tissue s were dissected. The placenta and fetus were then removed from the uterus. Placental tissues were stored for further experiments.

### 2.13 Systolic blood pressure (SBP) measurement

The animals were preheated in the healing chamber on the 6th, 12th, and 21st days. SBP was measured using the noninvasive tail-cuff method. The SBP measurement was repeated five times, and the average value for each animal was taken.

### 2.14 Proteinuria measurement

On the 6^th^, 12^th^, and 21^st^ day of pregnancy, urine was collected from the rats for 24 h to determine the urine protein. Then, the proteinuria was determined using a commercial kit (Sigma).

### 2.15 Histopathological observation

Rat placenta tissues’ pathological changes in each group were determined using Hematoxylin-eosin (HE) staining (Boster, Wuhan, China). The fixation of placental tissues was done using paraformaldehyde, and tissues were dehydrated using different concentrations of ethanol and then cleared with xylene. The tissues were then embedded in paraffin and cut into thin sections of 5 μm. After deparaffinization, the sections were stained with hematoxylin and eosin. The pathological changes were finally analyzed under an optical microscope (magnification, × 200).

### 2.16 Statistical analysis

Processing of all experimental data was done by SPSS 22.0 software. Data were presented as mean ± standard deviation (SD). The two-group comparison was made using a t-test. The comparison among multiple groups was made through a one-way analysis of variance (ANOVA). After ANOVA analysis, pairwise comparison was made using Tukey’s multiple comparisons test. *P* < 0.05 was considered statistically significant.

## 3 Results

### 3.1 SUF accelerates HTR8/SVneo cell proliferation

Pre-eclampsia (PE) is a prevalent pregnancy disease characterized by insufficient trophoblast cell migration (HTR8/SVneo). The study hypothesized that Sufentanil down-regulates the progression of pre-eclampsia via silencing microRNA-24-3p to target 11β-Hydroxysteroid Dehydrogenase Type 2. The study aimed to determine the effects of SUF on HTR8/SVneo cell viability, understand the effects of SUF on miR-24-3p and HTR8/SVneo cell proliferation, investigate the impacts of miR-24-3p mimicking on HTR8/SVneo cell progression, investigate if miR-24-3p targets HSD11B2 in PE and to understand the effects of SUF on HSD11B2 and HTR8/SVneo cell proliferation. Finally, the role of SUF in PE progression in vivo was investigated.

To determine the effects of SUF on PE, the human trophoblast HTR8/SVneo cells were treated with 5, 10, and 20 μM SUF. Cell viability was then determined with a CCK-8 assay. According to the results, treatment with 0–10 μM SUF led to the significant increase of cells in SUF-concentration-dependent manner, while the cells were significantly reduced following treatment with over 10 μM of SUF (Figure 1(a)). Next, colony formation was determined following treatment of the cells with 0, 5, 10, and 20 µM SUF. The results also confirmed significantly increased colony numbers following treatment with 5 and 10 µM SUF than the control. However, the colonies were significantly reduced after treatment with 20 µM SUF (Figure 1(b)). The transwell assays revealed a significantly increased cell migration and invasion after treatment with 5 and 10 µM SUF, which was inhibited following treatment with 20 µM of SUF (Figure 1(c,d)). The flow cytometry results confirmed significantly reduced apoptosis following treatment with 5, 10, and 20 µM of SUF compared to the controls, as shown in Figure 2(e). These observations confirmed that SUF induces the proliferation of HTR8/SVneo cells.

**Figure 1.** SUF inhibits miR-24-3p and accelerates HTR8/SVneo cell proliferation a-b: RT-qPCR detection of miR-24-3p; C: CCK8 test of HTR8/SVneo cell proliferation; d: Colony formation assay examination of HTR8/SVneo cells’ colony formation; e-f: Transwell detection of HTR8/SVneo cell invasion and migration; G: Flow cytometry test of HTR8/SVneo cell apoptosis. * *P* < 0.05, ** *P* < 0.01, *** *P* < 0.001 vs. the control; ^#^ *P* < 0.05, ^##^ *P* < 0.01, ^###^ *P* < 0.001 vs. the SUF + mimic NC. N = 3; Manifestation of the data in the figure was in the form of mean ± SD.

**Figure 2.** SUF accelerates HTR8/SVneo cell proliferation a: CCK8 detection of HTR8/SVneo cell proliferation; B: Colony formation assay test of HTR8/SVneo cells’ colony formation; c-d: Transwell examination of HTR8/SVneo cell invasion and migration; e: Flow cytometry test of HTR8/SVneo cell apoptosis. * *P* < 0.05, ** *P* < 0.01, *** *P* < 0.001. N = 3; Manifestation of the data in the figure was in the form of mean ± SD.

### 3.2 SUF inhibits miR-24-3p and accelerates HTR8/SVneo cell proliferation

To further verify the mechanisms of SUF on PE, RT-qPCR was used to determine miR-24-3p mRNA expressions in HTR8/SVneo cells treated with 0, 5, 10, and 20 µM SUF. The results showed significantly reduced miR-24-3p mRNA expressions in a SUF-concentration-dependent manner (Figure 2(a)). Next, miR-24-3p mRNA expressions were determined in the cells transfected with Sufentanil, Sufentanil +NC, or Sufentanil+ miR-24-3p or the control cells. The results confirmed a significant increase in miR-24-3p expression in Sufentanil+miR-24-3p compared to the controls (Figure 2(b)). The CCK-8 studies showed a significant drop in viability in the Sufentanil+miR-24-3p compared to the Sufentanil or Sufentanil+mimic-NC cells (Figure 2(c)). Similarly, the colony formation and transwell assays confirmed a significant reduction of cells in the Sufentanil+miR-24-3p compared to the Sufentanil or Sufentanil+mimic-NC cells (Figure 2(d-f)). However, the flow cytometry results confirmed significantly increased apoptosis in the Sufentanil+miR-24-3p than the Sufentanil or Sufentanil+mimic-NC cells (Figure 2(g)). These observations confirmed that SUF induces HTR8/SVneo cell proliferation through miR-24-3p-targeting.

### 3.3 MiR-24-3p mimicking suppresses s HTR8/SVneo cell progression

To investigate the role of miR-24-3p on HTR8/SVneo cells, the cells were transfected with mimic-NC, miR-24-3p mimic, inhibitor-NC, or miR-24-3p inhibitor. RT-qPCR was then used to determine miR-24-3p expression. The results confirmed significantly increased miR-24-3p expression in the miR-24-3p mimic compared to the miR-24-3p inhibitor and controls (Figure 3(a)). The CCK-8, colony formation, and transwell results confirmed significantly reduced cell viability (Figure 3(b)), cell colonies (Figure 3(c)), cell migration (Figure 3(d)), and cell invasion (Figure 3(e)) in miR-24-3p mimic compared to the miR-24-3p inhibitor and controls. The flow cytometry analysis results confirmed significantly increased apoptosis rate in the miR-24-3p mimic compared to the miR-24-3p inhibitor and controls (Figure 3(f)). These results confirmed that elevated miR-24-3p down-regulated the growth of HTR8/SVneo cells, while its repression had an opposite effect.

**Figure 3.** MiR-24-3p mimicking suppresses s HTR8/SVneo cell progression a: RT-qPCR detection of miR-24-3p; b: CCK-8 test of HTR8/SVneo cell proliferation; c: Colony formation assay examination of HTR8/SVneo cells’ colony formation; d-e: Transwell detection of HTR8/SVneo cell proliferation, invasion and migration; f: Flow cytometry test of HTR8/SVneo cell apoptosis. * *P* < 0.05, ** *P* < 0.01, *** *P* < 0.001 vs. the mimic NC; ^#^ *P* < 0.05, ^##^ *P* < 0.01, ^###^ *P* < 0.001 vs. the inhibitor NC. N = 3; Manifestation of the data in the figure was in the form of mean ± SD.

### 3.4 MiR-24-3p targets HSD11B2 in PE

To determine the association of miR-24-3p and HSD11B2 in PE, miR-24-3p mRNA expression was determined in the peripheral blood from healthy and PE-clinical samples. The results confirmed that miR-24-3p is significantly increased in the PE than in healthy tissues. However, HSD11B2 mRNA expression was significantly reduced in the PE than in healthy samples (Figure 4(a)). Rt-qPCR was then used to determine miR-24-3p and HSD11B2 expressions in miR-24-3p mimic, inhibitor-NC, miR-24-3p inhibitor, or mimic-NC transfected cells. The results confirmed significantly increased miR-24-3p but reduced HSD11B2 mRNA expressions in miR-24-3p mimic-transfected cells compared to the miR-24-3p inhibitor or control cells (Figure 4(b)).

**Figure 4.** MiR-24-3p targets HSD11B2 in PE a: RT-qPCR detection of miR-24-3p and HSD11B2 in 35 PE patients and healthy patients’ peripheral blood, *** *P* < 0.001 vs. the Health; B: RT-qPCR test of miR-24-3p and HSD11B2 in HTR8/SVneo cells, N = 3, ** *P* < 0.01, *** *P* < 0.001 vs. the mimic NC, ^##^ *P* < 0.01, ^###^ *P* < 0.001 vs. the inhibitor NC; c: Bioinformatics website starbase prediction of binding sites of miR-24-3p with HSD11B2; d: The luciferase activity assay verification of the binding of miR-24-3p with HSD11B2; E: RIP examination of the binding of miR-24-3p with HSD11B2; Manifestation of the data in the figure was in the form of mean ± SD.

The prediction of binding sites confirmed that miR-24-3p binds to HSD11B2 at the 3’-UTR region (Figure 4(c)). The dual-luciferase assay results also confirmed a significantly reduced luciferase activity in the WT-HSD11B2 cells transfected with miR-24-3p mimic compared to the mimic-NC cells (Figure 4(d)). Further, the RIP assays confirmed significantly increased enrichment in the Anti-Ago2 compared to Anti-G in both miR-24-3p and HSD11B2 that miR-24-3p bind with HSD11B2 (Figure 4(e)). These observations confirmed that HSD11B2 is a target of miR-24-3p.

### 3.5 SUF reverses the inhibitory effects of miR-24-3p on HTR8/SVneo cell proliferation

To determine the role and relationship between SUF and HSD11B2 in PE, RT-qPCR was used to analyze HSD11B2 mRNA expression in the cells treated with various concentrations of Sufentanil. The results demonstrated increasing HSD11B2 mRNA concentrations in a SU-dependent manner. Western blot experiments also confirmed significantly increasing HSD11B2 expression in a Sufentanil-dose-dependent manner (Figure 5(a)). Next, the HTR8/SVneo cells were transfected with oe-HSD11B2, oe-NC, oe-HSD11B2+ mimic-NC, oe-HSD11B2+ miR-24-3p mimic or the controls. The RT-qPCR was then used to determine mRNA expressions. According to the results, miR-24-3p mRNA expression was significantly increased in the cells transfected with oe-HSD11B2+ miR-24-3p mimic compared to the controls. According to the RT-qPCR and western blot results, the HSD11B2 expression was also significantly increased in the oe-HSD11B2, oe-HSSD11B2+ mimic-NC, and the oe-HSD11B2+ miR-24-3p mimic compared to the controls (Figure 5(b)).

**Figure 5.** SUF reverses the inhibitory effects of miR-24-3p on HTR8/SVneo cell proliferation a-b: RT-qPCR/WB test of miR-24-3p and HSD11B2; c: CCK-8 detection of HTR8/SVneo cell proliferation; d: Colony formation assay detection of HTR8/SVneo cells colony formation; e-f: Transwell examination of HTR8 /SVneo cell invasion and migration; G: Flow cytometry test of HTR8/SVneo cell apoptosis. * *P* < 0.05, ** *P* < 0.01, *** *P* < 0.001 vs. the oe NC or control; ^#^ *P* < 0.05, ^##^ *P* < 0.01, ^###^ *P* < 0.001 vs. the oe HSD11B2 + miR-24-3p mimic. N = 3; Manifestation of the data in the figure was in the form of mean ± SD.

The CCK-8, colony formation, and transwell experiments also confirmed significantly increased cell viability (Figure 5(c)), colony formation (Figure 5(d)), and cell migration and invasion (Figure 5(e-f)) in the oe-HSD11B2 and oe-HSD11B2+ mimic-NC groups compared to the oe-HSD11B2+ miR-24-3p mimic cells. However, the flow cytometry results confirmed a significantly reduced apoptosis in the oe-HSD11B2 and oe-HSD11B2+ mimic-NC groups compared to the oe-HSD11B2+ miR-24-3p mimic cells (Figure 5(g)). These observations confirmed that SUF accelerated HSD11B2 and reverses the suppressive effects of miR-24-3p on HTR8/SVneo cell progression.

### 3.6 SUF suppresses PE progression in vivo via miR-24-3p/HSD11B2 axis

The effects of SUF on the progression of PE in rats were further studied in *vivo* via the miR-24-3p/HSD11B2 axis. Systolic blood pressure (SBP) and 24-h proteinuria were determined on the 6^th^, 12^th^, and 21^st^ day of pregnancy. The fetal body weight was then determined after euthanasia. The SBP and proteinuria were significantly elevated in the PE group on day 12 and day 21. However, the SBP and proteinuria level was significantly reduced after treatment with Sufentanil in the PE+sufentanil group on both day 12 and day 21 (Figure 6(a,b)).

**Figure 6.** SUF suppresses PE progression in vivo via miR-24-3p/HSD11B2 axis a-b: Determination of rats’ SBP and 24 h proteinuria in different groups on the 6^th^, 12^th^ and 21^st^ d of pregnancy; c: Rats’ fetal weight in different groups; d: RT-qPCR detection of miR-24-3p and HSD11B2 of rat in each group; e: WB test of HSD11B2 of rats in each group; f: HE staining examination of placenta’s pathological changes of rats in each group (scale bar: 100 μm); *** *P* < 0.001 vs. the control; ^#^ *P* < 0.05, ^##^ *P* < 0.01, ^###^ *P* < 0.001 vs. the PE. N = 6; Manifestation of the data in the figure was in the form of mean ± SD.

Similarly, fetal weight was significantly elevated after treatment with SUF compared to the control and PE animals (Figure 6(c)). The relative miR-24-3p and HSD11B2 mRNA expression was then determined in normal pregnant mice, PE, or the PE+SU-treated animals. The results confirmed significantly increased miR-24-3p mRNA but reduced HSD11B2 mRNA expressions in the PE animals compared to the PE+ Sufentanil group (Figure 6(d)). The western blot assay also confirmed significantly reduced HSD11B2 proteins in the PE than the PE+ Sufentanil groups (Figure 6(e)). In PE rats, the placental tissue’s villi basement membrane was thickened to form a thrombus with placental hemorrhagic infarction. Pregnant mice’ placental villi cells in control were evenly distributed, the cell morphology was normal, and the tube wall was smooth. Additionally, PE rats’ pathology was ameliorated after SUF treatment (Figure 6(f)). Summarily, these results show that SUF restrained the progression of PE in rats via modulating the miR-24-3p/HSD11B2 axis.

## 4 Discussion

PE is characterized by an impaired invasion of trophoblast cells [18]. A critical pathology of PE is the disorder of maternal immune tolerance to the hemiallogeneic fetus, which is linked with an aberrant elevation of the four-transmembrane protein CD81 in trophoblast cells [4]. Additionally, the earlier the onset of PE, the higher the mean arterial pressure and urinary protein, the more severe the placental and fetal damage, while the trophoblast mitochondrial damage might act as different PE models’ joint terminal pathways [19]. Consequently, it is critical to understand the trophoblast function regulation mechanism to develop potential molecular biomarkers of PE treatment and early diagnosis. This research highlights a possible molecular mechanism of modulating trophoblast cell function. This study confirmed that a low concentration of SUF boosted trophoblast cell progression in *vivo* and in *vitro* via silencing miR-24-3p to accelerate HSD11B2, thereby constraining PE’s progression while the elevated concentration of SUF confirmed cytotoxicity.

Imperative labor analgesia can reduce pain and exert a critical action in ensuring the safety of mother and baby. Due to its stable hemodynamics and strong analgesic effect, SUF is broadly adopted in epidural labor and analgesic delivery [20]. Multiple reports have elucidated that SUF pretreatment and post-treatment have protective effects on PE parturients. For instance, spinal epidural anesthesia of combining with SUF is safer and more imperative for anesthesia management of PE patients [21]. SUF combined with bupivacaine can reduce the incidence of hypotension during cesarean section in severe PE patients [22].

Additionally, long-term epidural analgesia, including SUF, alleviates the labor pain in PE patients and immediately targets the pathogenesis of PE for operation [9]. Nevertheless, the latent mechanism of SUF targeting PE remains uncertain. The incidences of PE are associated with trophoblast dysfunction; hence it has been speculated that SUF might influence PE via modulating trophoblast cell function. In this study, HTR8/SVneo trophoblast cells were treated with three different concentrations of SUF. The results confirmed that SUF accelerated HTR8/SVneo cell progression in a concentration-dependent manner in the range of 0–10 μM. The progression of on HTR8/SVneo was reduced after over 10 μM. Besides, in *vivo* experimental results also confirmed that SUF restrained the progression of PE in rats, indicating that SUF has a latent therapeutic effect against PE.

Later, the molecular mechanism of SUF in PE treatment was explored. According to several studies, SUF mediates diverse cellular activities via modulating miRNA. For instance, SUF strengthens IκB-α via modulating the miR-129-5P/HMGB1 axis, thus suppressing the lipopolysaccharide-stimulated human bronchial epithelial cell apoptosis [23]. In this research, SUF restrained miR-24-3p, demonstrating that the action of SUF in PE might be linked with reduced miR-24-3p. Several reports have confirmed that miR-24-3p is elevated in the plasma of pregnant women with pregnancy-associated complications (like PE). Nevertheless, its specific function remains unknown [24,25]. In this research, miR-24-3p was increased in peripheral blood of PE patients. Repression of miR-24-3p accelerated trophoblast cell progression, while elevated miR-24-3p reversed the acceleration of SUF on trophoblast cell proliferation. SUF was shown to repress PE progression via inhibiting miR-24-3p. Additionally, miR-24-3p was negatively linked with HSD11B2, which was negatively modulated via miR-24-3p.

HSD11B2 is an enzyme that modulates local glucocorticoid (GC) [26]. Excessive exposure to GC during pregnancy is harmful to fetal development, while HSD11B2 acts as the GC barrier during this process, protecting the fetus [27]. The activity of HSD11B2 in serum is elevated during normal pregnancy [28]. PE reduces the activity of HSD11B2, leading to increased fetal GC [29]. Consequently, targeting HSD11B2 might be the novel strategy for PE therapy. In this research, HSD11B2 was reduced in peripheral blood of PE patients, and it was increased following the treatment with SUF. Additionally, increased HSD11B2 turned around the effect of upregulated miR-24-3p, enhancing trophoblast cell proliferation.

## 5 Conclusion

In conclusion, SUF accelerates the proliferation of HTR8/SVneo cells via miR-24-3p inhibition. Further, SUF elevates HSD11B2 by targeting miR-24-3p, accelerating the progression of trophoblast cells, thereby constraining PE progression. Finally, SUF suppresses PE progression in vivo through miR-24-3p/HSD11B2 axis. The use of SU to inhibit miR-24-3p may provide a novel idea in the development of a biomarker for PE therapy. In addition, this investigation provides a future direction that mechanisms targeting the blocking of HSD11B2 could be effective therapeutic approaches against PE.

## Supplementary Material

Supplemental Material
